This article has been retracted.

# Green transition in manufacturing: Dynamics and simulation

**DOI:** 10.1371/journal.pone.0280389

**Published:** 2023-01-20

**Authors:** Lin Lu, Xue Su, Song Hu, Xiaochun Luo, Zhangzheyi Liao, Yuelin Ren, Kai Kang, Beibei Li

**Affiliations:** 1 School of Economics and Management, Guangxi Normal University, Guilin, China; 2 School of Business Administration, Guizhou University of Finance and Economics, Guiyang, China; 3 Henan Polytechnic, Zhengzhou, China; 4 School of Economics and Management, Nanjing University of Aeronautics and Astronautis, Nanjing, China; 5 School of Economics and Management, Heilongjiang Bayi Agricultural University, Daqing, China; Shenzhen University, CHINA

## Abstract

Under the dual background of global industrial value chain and low-carbon emission reduction, the green transformation and upgrading of the manufacturing industry is an important way to promote production and promote sustainable economic development. Considering that the green transformation of the manufacturing industry is a typical complex adaptation system, based on the intrinsic relationship between the dynamic theory and the green transformation of the manufacturing industry, this paper takes the endogenous variable of the transformation of manufacturing enterprises as the entry point, simulates the transformation of new and old dynamic energy of green transformation, and explores the mechanism of green transformation and upgrading of manufacturing industry and the conversion process. According to the model, it is concluded that the green transformation of manufacturing enterprises is the result of the multi-stage transformation of enterprises. In this process, the change inertia overcomes old dynamic inertia and promotes the new dynamic to gradually replace the old dynamic. At the end of the article, specific suggestions are given to promote the green transformation of manufacturing enterprises from the aspects of ideology, policy support, digital empowerment, financial service guarantee system and communication and cooperation.

## 1. Introduction

Environmental issues have become an important problem that needs to be solved urgently in countries around the world, among which greenhouse gas emissions pose a serious threat to human survival and sustainable social and economic development [1], and governments attach great importance to environmental protection and green development, formulate national sustainable development strategies [2], and introduce a series of emission reduction measures and policies [3], including the UK Climate Change Agreement, the German Climate Protection Plan 2050, and Made in China 2025.

Manufacturing drives economic growth while also becoming a major source of greenhouse gas emissions [4], and its high-investment, energy-intensive, and polluting economic developments place a serious burden on the natural environment [5]. As the most important component of the industry, the green development of the manufacturing industry is crucial to achieving the dual goals of carbon emissions (carbon peak and carbon neutrality) [6], so it is necessary to improve product quality, introduce or develop energy-saving and environmental protection technologies, and achieve green transformation and upgrading [7]. In particular, the manufacturing industry is embedded in developing countries downstream of the global value chain, resulting in a large number of carbon emission cost pressures [8], under the pressure of re-industrialization in developed countries and low-cost industrial transfer in developing countries [6], green transformation and upgrading needs to be more urgent [9], for this reason, a large number of scholars focus on the green transformation and upgrading of manufacturing in developing countries, and carry out relevant research from many aspects.

The research related to the green transformation and upgrading of management and manufacturing industry mainly includes three aspects, namely the evaluation system, driving factors, and transformation and upgrading paths. The unmeasurable green level of the manufacturing industry cannot be transformed and improved [10], and by clearly assessing the green status of the manufacturing industry, it can provide a direction and path for the green transformation of the manufacturing industry. Low-carbon green is a comprehensive concept, involving the measurement of multiple indicators, for this reason, including Qu [11], Pan [12], Peng [13], Yin [14] and many other scholars to build a manufacturing green growth and innovation performance evaluation system, to identify the green performance of the manufacturing industry, and to propose targeted transformation and upgrading measures. In order to avoid the error caused by decision subjectivity, many scholars have tried to optimize the index model in recent years, and Wang combined the fuzzy hierarchy analysis method and the fuzzy ideal solution similar sorting technique to propose a hybrid multi-criteria decision model [15]. Based on the improved particle swarm optimization algorithm, Wang constructed the greenness evaluation system of the equipment manufacturing industry [16]. Considering that intelligence is an important boost to the green transformation and upgrading of the manufacturing industry [17], Yin constructed a performance evaluation model for digital green innovation in the manufacturing industry, including pressure systems, state systems and response systems [18].

Although green development has become the trend of the times [19], in general, green transformation as a change will impose additional costs on enterprises, which directly hinders the independent transformation of enterprises [20], Sajid said that "cost reduction" and "government support" are the main drivers of green innovation time in the manufacturing industry of developing economies [21]. The ideal green transformation cost can be paid by the money saved by green manufacturing [22], but considering the uncertainty of risk returns, external factors such as managers’ risk preferences, and internal factors such as corporate assets, driving the green transformation and upgrading of the manufacturing industry cannot rely solely on the company’s own transformation willingness.

As an effective means for the government to promote the green transformation of enterprises, government regulations have become the focus of many scholars’ research [23]. Constrained by carbon tax [24], cap and trade [25] and uncertainty of closed-loop logistics [26, 27], many scholars build quantitative models to find the optimal corporate profits and social welfare [28–30]. With sustainable innovation and green dynamic capabilities as the mediator [31], environmental regulations affect the sustainable performance of enterprises [32]. Enterprises with more green innovation dynamic will obtain higher sustainable benefits [33]. Lu further developed the research results, and believed that environmental regulation mainly improves financial performance through green process innovation rather than green product innovation [34]. Lei studied the impact of three types of environmental regulations on the green transformation and upgrading of the manufacturing industry [35], Zhang focused on the specific incentive effect of environmental technical standards, which is a command-controlled environmental regulation [36], and some scholars focused on the influence mechanism of trade comparative advantages under environmental regulations [37], green technology innovation [38, 39], and resource endowments [40].

Green transformation is the result of a complex impact. There are obvious differences in the impact of government regulations on enterprise innovation transformation in an uncertain environment [41, 42]. The lack of detailed provisions [43] and the lack of low-carbon performance of local governments [44] may also lead to a decline in the effect of environmental regulations. For this reason, some scholars explored ways to optimize environmental regulatory constraints. Pacces said that standardization of environmental sustainability disclosure is an important means to curb enterprises’ greenwashing behavior [45]. Esty believed that the standard models of environmental information regulation are ill-equipped to address the information needs of today’s investment community. He suggested a new design of environmental information regulation capable of harnessing mainstream investor interest in sustainability [46].

In the context of extensive digitalization in economy and society, sustainability is closely linked with digital transformation [47]. As an efficient tool capable of handling massive and complex data, digitalization has attracted extensive attention from scholars. A large number of research results show that digitalization has promoted the potential and performance of sustainable transformation [48–50] through changes in waste management [51, 52], pollution control [53, 54], sustainable production [55, 56] and other fields. Some scholars said that digitalization does not directly improve energy efficiency. Townsend believed that digitalization is an indirect way to achieve sustainable transformation of enterprises by promoting circular economy [57]. Jones also agrees with this view. He studies the enterprise reports of leading companies in digital transformation and believes that supporting and promoting the circular economy is a great opportunity for digitalization to affect sustainable development [58]. Tavoletti believes that digitalization will stimulate enterprises to transform their business models to maintain competitiveness [59].

In addition, scholars also explored the impact mechanism of management vision [60], employee expectations [61], organizational barriers [62], management model [63], industrial resource aggregation [64] and market demand and orientation [65–69], and tried to explore the internal and external green transformation dynamic energy of enterprises. Yang said that intelligent manufacturing, market demand and fixed asset investment are also important sources of power for the transformation and upgrading of the manufacturing industry [70], Song analyzed the impact mechanism of high-tech industrial agglomeration, and believed that it has a significant role in promoting the green transformation of manufacturing in the medium term of industrialization and economically underdeveloped areas [71], and Syed tested the impact of manufacturing and logistics industry cooperation on total factor green productivity [72]. Kazemargi emphasized the leading and coordinating role of core companies in innovation practice from the perspective of supply chain [73].

The research results on the transformation path of the manufacturing industry are relatively weak, Wang [74] and Yang [75] have proposed three upgrading paths: unilateral, leapfrog and jumping, and Du said that green technology innovation and industrial structure upgrading are important paths for green transformation and upgrading [76]. Dong proposed a parallel transformation and upgrading path from the industrial level, the element level and the institutional level [77]. On this basis, Zhang also proposed to build a green consumption system to achieve the active transformation of the manufacturing industry [78]. Lu focused on the transformation and upgrading path of small and medium-sized manufacturing enterprises, and discussed the obstacles and measures for upgrading in the path [79]. In addition to relying on the innovative research and development and reform of manufacturing enterprises themselves, some scholars have turned their goals to external resources to achieve more efficient transformation and upgrading. Xu believes that mergers and acquisitions are a strong boost to the green transformation of traditional manufacturing [80]. Some scholars have proposed that deep industrial integration is the key to green transformation and upgrading [81], and industrial integration can also indirectly affect the improvement of energy efficiency by expanding industrial scale and optimizing factor structure [82], Meng will specifically look at the production and service industry and manufacturing industry, and found that collaborative agglomeration and carbon emission intensity show an inverted n-shaped nonlinear relationship, and there is obvious heterogeneity in different sub-industries [83].

Looking at the existing research, the first is to analyze the influencing factors promoting the green transformation of the manufacturing industry from the macro perspective of innovation and policy, and lack of phased and evolutionary research on the green transformation process of the manufacturing industry; The second is to focus on the impact of exogenous environmental factors and ecological factors on the green transformation and upgrading of the manufacturing industry, and rarely consider the impact and promotion of endogenous variables on its transformation, and the third is mostly qualitative research, lack of necessary quantitative research, and poor explanatory power. Considering that the transformation and upgrading of the manufacturing industry is a process, it is necessary to understand the influence mechanism of the driving factors from the overall perspective, therefore, it is necessary to build a quantitative model that can quantitatively simulate the green transformation of the manufacturing industry, analyze the influence mechanism of internal and external factor variables in the transformation process, expose the transformation path and evolution process, and provide scientific guidance for the current green transformation and upgrading of the manufacturing industry.

The orderly transformation of old and new dynamic energy is the internal power to promote industrial transformation and upgrading [84]. When the old dynamic energy develops to a certain stage, it will inevitably weaken, and new dynamic energy will inevitably emerge to adapt to the new development pattern [85]. At the moment when green development has become the international mainstream, the replacement of old dynamic energy by new dynamic energy has become an important feature of green transformation of manufacturing enterprises. To promote high-quality development of manufacturing industry, it is necessary to get through the key nodes of the transformation of new and old dynamic energy of manufacturing industry [86]. Some scholars said that the industry will undergo radical changes when facing great threats [87], while incremental changes cannot bring about complete changes when facing climate problems [88]. Copani said that the upgrading of the most sustainable manufacturing product service system needs more radical changes [89]. However, considering that incremental innovation has higher Institutional attractiveness than radical innovation, and faces fewer systematic obstacles [90], the feasibility of the radical industrial green transformation strategy has also been questioned. Shi made a comprehensive consideration and believed that industrial upgrading is the result of the synergy of gradual and radical changes [91].

Taking the endogenous variable of manufacturing industry change as the starting point, this paper uses dynamic theory to analyze the evolution process of green transformation of manufacturing industry and its key driving factors, and reveals the evolution mechanism and trajectory of green transformation of manufacturing industry. The contribution of this article includes two aspects. The first is the innovative use of dynamic model, and taking into account the influence on endogenous variables in the green transition process, the dynamic evolution process between the stages is reflected by vectors, providing a visual quantitative simulation model for further analysis of the green transition path and mechanism of action. Secondly, the new and old dynamic energy functions and transformations of the green transformation process of the manufacturing industry are analyzed in stages, the mechanism and dynamic evolution process of the transformation of the new and old dynamic energy of the manufacturing industry are revealed, and the relevant suggestions for the green transformation of the manufacturing industry are proposed at the end.

## 2. The relationship between kinetic theory and the green transformation of manufacturing industry

The green transformation of manufacturing industry is a special manifestation of manufacturing transformation and upgrading, from the internal mechanism, there is an alternation of new and old dynamic energy in this process, in which the alternating change between new dynamic energy and old dynamic energy and the interaction relationship between related variables in the theory of energy transfer dynamics in physics are very consistent. Based on the dynamic theory in physics, this paper compares the movement of particles in an inertial and non-inertial frame with the mechanism of different degrees and different aspects of enterprise changes on the transformation process of new and old dynamic energy of enterprises. The centroid in the frame of reference in physics represents the leading manufacturing industry (hereinafter referred to as MRE), and the representative enterprise is the reference object of other enterprises in the manufacturing industry, and the representative enterprise is recorded as G. The mass point *m*_*i*_ represents a firm in the industry. Let the angular velocity of rotation of the center of mass $\vec{\omega_{c}}$ and the angular acceleration of rotation of the center of mass $\vec{\omega_{c}}$ correspond to the change ability of MRE behavior pattern $\vec{BR_{MRE}}$ and MRE change trend $\vec{TR_{MRE}}$ respectively, the greater the angular velocity of rotation, the greater the magnitude and strength of MRE change, the greater the acceleration, the smaller the path dependence of MRE change, the longer the trend and direction of change. The angular velocity of rotation can reflect the characteristics and movement of MRE change to a certain extent. $\vec{r_{o^{\prime }}}$ indicates the position vector of non-inertial reference system relative to the static system, reflecting the change of MRE before and after the transformation of old and new dynamics; $\vec{r^{\prime }{}_{c}}$ indicates the bit vector of center of mass c relative to the point, which can reflect the development level of MRE change; the speed of center of mass $\vec{v_{MRE}}$ and acceleration of center of mass $\vec{a_{MRE}}$ reflect the ability of MRE strategic change and behavioral pattern change. The faster the velocity of the center of mass, the stronger the MRE change ability; indicates the position vector of any mass point in the mass point group relative to the non-inertial reference system, which can reflect the change ability of an ordinary enterprise in the manufacturing industry relative to the MRE change level.

A diagram of the relationship between the action of the variables of kinetic theory is shown in Fig 1.

**Fig 1:** Momentum theorem for mass points in general non-inertial systems.

According to the second law of Newtonian mechanics and the momentum theorem, angular momentum theorem and dynamic energy theorem of the group of non-inertial system mass points, it is used to describe the process mechanism of green transformation of manufacturing industry and the key driving elements in it. In this paper, the green transformation process of manufacturing enterprises is divided into three different stages: in the first stage, the old dynamic energy still dominates the operation of enterprises; in the second stage, both the old dynamic energy and the new dynamic energy play a joint role in the upgrading evolution of enterprises; in the third stage, the new dynamic energy dominates and plays a major role in the upgrading evolution of enterprises, and in this stage, the new dynamic energy has basically replaced the old dynamic energy. Each different stage of the old and new dynamic energy momentum size shows the stage characteristics, the trend of the old and new dynamic energy of enterprises is shown in Fig 2.

**Fig 2:** Change of green transformation momentum in manufacturing industry at different stages.

This control relationship reflects to a certain extent the mechanism of action and dynamic evolution process of manufacturing enterprises in the process of green transformation. A variety of different variables are involved in this process, and the interaction relationship between variables can also be reflected by the interaction relationship of forces in kinetic theory. The specific relationships and the correspondence between variables are shown in Table 1.

**Table 1:** Cross-relationship between green transformation of manufacturing industry and kinetic theory.

Designation	The space of motion constituted by the set of mass points *m*_*n*_		The space of manufacturing enterprise group composition	
Center-of-mass motion parameter setting	O − XYZ is the static inertial reference system; O′ − XYZ is the non-inertial reference system moving with respect to O at moment t; c : center of gravity M : Total mass of the system of mass points; $\vec{v_{c}}$ : Velocity of Mass $\vec{a_{c}}$ : acceleration of the center of mass $\vec{\omega_{c}}$ : Angular velocity of rotation of the center of mass $\vec{u_{c}}$ : Angular acceleration of center of mass rotation $\vec{r_{c}}$ : The position vector of the center of mass C with respect to the o− system		O − XYZ for manufacturing companies to upgrade the frame of reference; O′ − XYZ is the reference frame for the change in the old and new dynamics of manufacturing enterprises at moment t; O′ : The transformation of old and new dynamic energy occurring in MRE at moment t K : Collection of original resources of all companies in the industry $\vec{SR_{MRE}}$ : MRE Strategic Change Capability $\vec{BR_{MRE}}$ : MRE Behavior Model Change Capability $\vec{TR_{MRE}}$ : MRE Change Trends $\vec{WR_{MRE}}$ : MRE Change Disruption Degree $\vec{LR_{MRE}}$ : MRE Change Development Level	
Mass settings and parameters	m : The mass of the mass point *m*_*i*_ $\vec{v}$ : Velocity of the mass *m*_*i*_ $\vec{a}$ : Acceleration of the mass *m*_*i*_ $\vec{a_{n}}$ : The normal acceleration acting on the mass *m*_*i*_ $\vec{a_{t}}$ : Tangential acceleration for mass m_i_ $\vec{F}$ : The combined external force acting on the mass *m*_*i*_ $\vec{F_{n}}$ : The normal force acting on the mass *m*_*i*_ $\vec{F_{t}}$ : The tangential force acting on the mass *m*_*i*_		k : Collection of resources for manufacturing company G $\vec{SR}$ : Manufacturing companies G existing strategic change capabilities $\vec{BR}$ : Behavioral model change capability of manufacturing company G $\vec{IR_{gra}}$ : Progressive change intensity of manufacturing company G $\vec{RR_{rad}}$ : The intensity of radical change in manufacturing company G $\vec{ND}$ : The new dynamics of manufacturing company G $\vec{ND_{n}}$ : The new dynamics of resources for manufacturing companies G $\vec{ND_{t}}$ : New market dynamics for manufacturing company G	
Mass change inertia parameter setting	$\vec{f_{1}}$ : The implicated inertial force of the mass *m*_*i*_	$\vec{f_{1}}$ : The translational inertia force of the mass *m*_*i*_ $\vec{f_{t}}$ : The tangential inertia force of the mass *m*_*i*_ $\vec{f_{s}}$ : The inertial centrifugal force of the mass *m*_*i*_	$\vec{I_{G}}$ : Consistent inertia of G versus MRE upgrade changes in manufacturing companies	$\vec{I_{gra}}$ : Progressive change inertia $\vec{I_{rad}}$ : Radical change inertia $\vec{I_{str}}$ : Internal structural change inertia
The old dynamic energy inertia parameter setting of the mass	$\vec{f_{c}}$ : Koch Practice		$\vec{I_{OK}}$ : Manufacturing companies G relative to MRE upgrade changes old momentum inertia	
Parameter setting for mass momentum	$\vec{r}$ : The position vector of the mass m_i_ with respect to the O- system $\vec{r^{\prime }}$ : The position vector of the mass m_i_ with respect to the O′ - system $\vec{P}$ : The momentum of the mass m_i_ with respect to the O- system $\vec{P^{\prime }}$ : The momentum of the mass m_i_ with respect to the O′- system		$\vec{LSR}$ : Strategic change level vector of manufacturing company G relative to O-system $\vec{LSR^{\prime }}$ : Vector of strategic change level of manufacturing firm G relative to O′-system $\vec{OKE}$ : Manufacturing firm G relative to the old dynamic momentum of the O-system $\vec{OKE^{\prime }}$ : Manufacturing firm G relative to O′-system old dynamic momentum	

There is a certain quantitative relationship between the motion of the mass point and the momentum of the mass point, the inertial force on the mass point and the external force acting on the mass point, etc. This quantitative relationship can reflect to a certain extent the mechanism of manufacturing change in the process of green transformation and the change process of new dynamic energy replacing old dynamic energy. The specific quantitative relationship is shown in Table 2.

**Table 2:** Interaction relationship between variables in the process of green transformation of manufacturing.

Designation	Mechanical relations in theoretical mechanics	The interaction between the intensity of change in manufacturing, the momentum of old dynamic energy, the strength of new dynamic energy and inertia in the process of changing old and new dynamic energy	Formula number
Static system	$\vec{F}=\vec{F_{n}}+\vec{F_{t}}$	$\vec{ND}=\vec{ND_{n}}+\vec{ND_{t}}$	(1)
	$\vec{F}=m\times \vec{a}=m\times \frac{d\vec{v}}{dt}$	$\vec{ND}=k\times \vec{BR}=k\times \frac{d\vec{SR}}{dt}$	(2)
	$\vec{p}=m\times \vec{v}=m\times \frac{d\vec{r}}{dt}$	$\vec{OKE}=k\times \vec{SR}=k\times \frac{d\vec{LSR}}{dt}$	(3)
	$\Delta \vec{p}=\int \vec{F}\times dt$	$\Delta \vec{OKE}=\int \vec{ND}\times dt$	(4)
Relationship between variables	$\vec{r}=\vec{r_{O^{\prime }}}+\vec{r^{\prime }}$	$\vec{LSR}=\vec{LR_{MRE}}+\vec{LSR^{\prime }}$	(5)
	$\vec{v}=\vec{v_{O^{\prime }}}+\vec{v^{\prime }}$	$\vec{SR}=\vec{SR_{MRE}}+\vec{BR}$	(6)
	$\vec{a}=\vec{a_{O^{\prime }}}+\vec{a^{\prime }}$	$\vec{BR}=\vec{BR_{MRE}}+\vec{BR^{\prime }}$	(7)
Non-inertial system	$\vec{f_{G}}=\vec{f_{l}}+\vec{f_{t}}+\vec{f_{n}}$	$\vec{I_{G}}=\vec{I_{l}}+\vec{I_{t}}+\vec{I_{n}}$	(8)
	$\vec{f_{l}}=-m\times \vec{a_{c}}$	$\vec{I_{gra}}=-k\times \vec{BR_{MRE}}$	(9)
	$\vec{f_{t}}=-m\times \vec{u_{c}}\times \vec{r_{c}}$	$\vec{I_{rad}}=-m\vec{TR_{MRE}}\times \vec{LR_{MRE}}$	(10)
	$\vec{f_{n}}=-m\times \vec{\omega_{c}}\times \left(\vec{\omega_{c}}\times \vec{r_{c}}\right)$	$\vec{I_{str}}=-k\times \vec{TR_{MRE}}\times \left(\vec{TR_{MRE}}\times \vec{LR_{MRE}}\right)$	(11)
	$\vec{f_{c}}=-2m\times \vec{\omega_{c}}\times \vec{v_{c}}$	$\vec{I_{OK}}=-2k\times \vec{TR_{MRE}}\times \vec{SR_{MRE}}$	(12)
	$\vec{P^{\prime }}=\vec{P}-m\times \vec{v_{c}}$	$\vec{OKE^{\prime }}=\vec{OKE}-K\times \vec{SR_{MRE}}$	(13)
	$\Delta \vec{P^{\prime }}=\int \left(\vec{F}+\vec{f_{G}}+\vec{f_{c}}\right)\times dt$	$\vec{OKE^{\prime }}=\int \left(\vec{ND}+\vec{I_{G}}+\vec{I_{OK}}\right)\times dt$	(14)

## 3. Manufacturing green transformation dynamics model

In this paper, the green transformation process of manufacturing industry is divided into three different stages. In the first stage, the old dynamic energy still occupies the dominant position in the operation of manufacturing enterprises; in the second stage, both old and new dynamic energy play a role in the upgrading and evolution process of manufacturing enterprises; in the third stage, new dynamic energy dominates and plays a major role in the upgrading and evolution process of manufacturing enterprises, and new dynamic energy has basically replaced old dynamic energy in this stage. Each different stage of the new and old dynamic energy momentum size shows the characteristics of the stage, this contrast relationship to a certain extent reflects the role of the manufacturing industry in the process of the old and new dynamic energy conversion mechanism and dynamic evolution process. There are many different variables involved in this process, and the interaction relationship between variables can also be reflected by the interaction relationship of forces in kinetic theory.

### 3.1. Changes in green transformation of manufacturing enterprises in the stage of dominance of old dynamic energy

Manufacturing firms are biased to transform and improve the original old dynamic energy, but will not go into substantial change and implement replacement of the old dynamic energy. In this stage, MRE has not yet implemented obvious changes, and this paper corresponds the upgrading of manufacturing firms in this period with the static system in theoretical mechanics. Taking as the static reference system, at the initial moment of this stage, the strategic change ability of manufacturing enterprises is, the behavioral model change ability of manufacturing enterprises is, the new dynamic energy of production factors of manufacturing enterprises is, and the old dynamic energy momentum of manufacturing enterprises is. This stage of green transformation of manufacturing enterprises is mainly reflected in the improvement or optimization of the old dynamic energy of manufacturing enterprises, so that the old dynamic energy can keep the same pace with the MRE changes, the moment of the end of this stage, the inertia force of the old dynamic energy is enhanced, that is, the inertia force of the old dynamic energy is changed from the original, the behavior mode change ability of manufacturing enterprises becomes, manufacturing enterprises to behavior change mode, according to the kinetic theory, the momentum The greater the inertia is also greater, according to the formula in Table 2, there is

$$\vec{OKE_{1}}=\vec{BR_{1}}\times k-\vec{ND_{0}}\times t-\int_{t_{0}}^{t_{1}}\left[\vec{ND_{n}}+\vec{ND_{t}}\right]dt-\vec{OKE_{0}}$$ (15)

According to the formula of vector (reflecting the magnitude of the force) in theoretical mechanics, the angle of rotation of the strategic change capability of a manufacturing company around the O system is Ω_1_, Then the strategic change level vector $\vec{LSR}$ of manufacturing companies is $\vec{LSR}=t\vec{SR_{1}}\text{cos}\;\theta_{1}$; The angle of rotation of the manufacturing firm’s behavioral model change capability around the O-system is θ_2_, The manufacturing firm behavior model change vector $\vec{LBR}$ is $\vec{LSR}=t\vec{SR_{1}}\text{cos}\;\theta_{1}$

$$\vec{LBR}={\text{sin}}^{2}\;\theta_{2}+\text{cos}\;\Omega_{2}$$ (16)

$\vec{ND}$ denotes the factor dynamic energy of manufacturing firms, Let the enterprise production factor dynamic energy vector be $\vec{LBR}$, The dynamic energy of the production factor is rotating around the O system at an angle of Ω_3_, The manufacturing company originally had a state of old dynamic energy as a force of angle, Then we have

$$\vec{LND}={\text{sin}}^{2}\;\theta_{3}+\text{cos}\;\Omega_{3}$$ (17)

As far as the change of MRE is concerned, the reference system of MRE evolves from O − XYZ to O′ − XYZ at moment t. The motion state of the center of mass O represents the state and degree of the old and new dynamic energy transition of MRE. At a certain moment t, $\vec{SR_{MRE}}$ represents the MRE’s strategic change capacity, let the MRE’s MRE change level vector (i.e., size) at this moment be $\vec{LSR_{\text{c}}}$ and the angle of rotation of the MRE’s strategic change effort around the O′ system be *δ*_1_. Then we have

$$\vec{LSR_{MRE}}=\text{t}\vec{SR_{MRE}}\times \text{arccos}\;\delta_{1}$$ (18)

$\vec{BR_{MRE}}$ represents the behavior pattern change ability of MRE, and let the angle of its winding around the O′-system be *δ*_4_, then the behavior pattern change level vector of MRE is

$$\vec{LBR_{MRE}}=\vec{BR_{MRE}}\times \text{tan}\;\delta_{4}$$ (19)

$\vec{TR_{MRE}}$ reflects the trend of MRE change, and according to the formula of center of mass and angular velocity, there is

$$\vec{TR_{MRE}}=\frac{\varphi }{t}$$ (20)

where *φ* denotes the angular magnitude of the rotation of the mass around the origin of the system, in units of rad/s.

$\vec{LWR_{MRE}}$ denotes the magnitude of the destructive degree brought by the MRE change, and let the angle of the MRE change destructive force moving around the O′-system be *δ*_5_, then

$$\vec{LWR_{MRE}}=\frac{d\vec{TR_{MRE}}}{dt}=\frac{\varphi }{t^{2}}$$ (21)

According to equation (2) in Table 2, the size of the old dynamic inertia of the manufacturing firm at any given moment has

$$\vec{OKE}=k\times \frac{d\vec{LSR}}{dt}=k\vec{SR}$$ (22)

The behavioral model change of manufacturing companies in the first phase enhances the old dynamic energy momentum of manufacturing companies.

$$\vec{BR_{1}}=P_{a}^{\alpha }R_{a}^{\alpha }>\vec{SR_{1}}=P_{b}^{\alpha }R_{b}^{\alpha }$$ (23)

where *P*_*a*_ denotes the probability that the manufacturing firm will implement behavioral model change in the first stage; *P*_*a*_ denotes the probability that the manufacturing firm will achieve strategic change. From Eq (23), it is clear that manufacturing firms are likely to adopt behavioral model change more in the first stage.

### 3.2. The old and new dynamics work together in the process of green transformation and upgrading of manufacturing enterprises stage

At the initial moment *t*_1_ of this stage, the old dynamic energy momentum of manufacturing enterprises becomes $\vec{OKE_{1}}$, the strategic change capability of manufacturing enterprises at the end moment *t*_2_ of this stage should be enhanced to $\vec{SR_{2}}$, and the relative strategic change capability of manufacturing enterprises relative to the MRE change level is $\vec{BR_{2}}$; the behavioral pattern change capability of manufacturing enterprises themselves at this moment is enhanced to $\vec{SR^{\prime }{}_{2}}$, and the behavioral pattern change capability relative to MRE is $\vec{BR^{\prime }{}_{2}}$; manufacturing firm’s new dynamic energy of production factors at this time is $\vec{ND_{1}}$. According to the theoretical mechanics formula there is new dynamic energy.


$$\begin{array}{l} \vec{ND_{1}}+\vec{ND_{t}}={\left[k\times t\times \vec{BR^{\prime }{}_{2}}-\vec{ND_{1}}\times t\right]}^{\prime }+k\times \vec{BR_{MRE}}\\ ={\left[k\times t\times \vec{SR^{\prime }{}_{2}}-\vec{ND_{1}}\times t-\vec{OKE^{\prime }{}_{1}}\right]}^{\prime }+k\times \vec{BR_{MRE}} \end{array}$$ (24)

As can be seen from the above equation, the stronger the relative strategic change ability of manufacturing enterprises, beyond the average level of MRE, and at this time the role of new dynamic energy of production factors, the change of representative enterprises in the industry to other manufacturing enterprises to implement change to play a certain demonstration and incentive role. The strategic change capabilities of the second stage manufacturing companies are

$$\begin{array}{l} \vec{SR^{\prime }{}_{2}}=\frac{\vec{ND_{1}}\times t+\vec{LR}+\int_{t_{1}}^{t_{2}}\left[\vec{ND_{n}}+\vec{ND_{t}}-k\times \vec{BR_{MRE}}\right]\times dt}{k}\\ =\frac{\vec{ND_{1}}\times t+\frac{{\left[\sum_{j=1}^{m}F_{ij}-F_{i}^{+}\right]}^{\frac{1}{2}}}{\text{min}{\left[\sum_{j=1}^{m}F_{ij}-F_{i}^{+}\right]}^{\frac{1}{2}}}/\frac{{\left[\sum_{j=1}^{m}F_{ij}-F_{i}^{-}\right]}^{\frac{1}{2}}}{\text{max}{\left[\sum_{j=1}^{m}F_{ij}-F_{i}^{-}\right]}^{\frac{1}{2}}}+\int_{t_{1}}^{t_{2}}\left[k\times \frac{d\vec{SR}}{dt}-k\times \vec{BR}\right]\times dt}{k} \end{array}$$ (25)

$$\begin{array}{l} \vec{BR^{\prime }{}_{2}}=\frac{\vec{ND_{1}}\times t+\int_{t_{1}}^{t_{2}}\left[\vec{ND_{n}}+\vec{ND_{t}}-k\times \vec{BR_{MRE}}\right]\times dt}{e}\\ =\frac{\vec{ND_{1}}\times t++\int_{t_{1}}^{t_{2}}\left[k\times \frac{d\vec{SR}}{dt}-k\times \vec{BR}\right]\times dt}{e} \end{array}$$ (26)

$\vec{SR^{\prime }{}_{2}}>\vec{BR^{\prime }{}_{2}}$, It can be seen that manufacturing companies in the second stage of strategic change is more powerful than behavioral model change.

### 3.3. The new dynamic energy of manufacturing enterprises dominates and has basically replaced the old dynamic energy stage

At the initial moment *t*_2_ of this stage, the strategic change ability of manufacturing enterprises is $\vec{SR_{2}}$, the behavioral model change ability of manufacturing enterprises is $\vec{BR_{2}}$, the new dynamic energy of production factors of manufacturing enterprises increases to $\vec{ND_{2}}$, and the old dynamic energy momentum of manufacturing enterprises is $\vec{OKE_{2}}$. In this stage, the radical change intensity of manufacturing enterprises has increased to a large extent, and the large and more radical change makes the new dynamic energy of manufacturing enterprises The inertia of change increases to a large extent, gradually overcoming the inertia of old dynamic energy, and the level of change catches up with the level of change of MRE. At any moment t_3_ of this stage, the strategic change ability of manufacturing enterprise relative to MRE is $\vec{SR^{\prime }{}_{3}}$, the behavioral pattern change ability relative to MRE is $\vec{BR^{\prime }{}_{3}}$, the old dynamic energy momentum of manufacturing enterprise is $\vec{OKE_{3}}$, and the new dynamic energy of production factor of manufacturing enterprise is $\vec{ND_{3}}$. According to the theoretical mechanics formula in Table 2, there are new dynamic energy of human resources $\vec{ND_{n}}$ and new dynamic energy of market $\vec{ND_{t}}$.


$$\begin{array}{l} \vec{ND_{n}}+\vec{ND_{t}}={\left[k\times t\times \vec{BR^{\prime }{}_{3}}-\vec{ND_{2}}\times t\right]}^{\prime }+k\times \vec{BR_{MRE}}+k\times \vec{WR_{MRE}}\times \vec{LR_{MRE}}\\ +k\times \vec{TR_{MRE}}\times \left(\vec{TR_{MRE}}\times \vec{LR_{MRE}}\right)+2k\times \vec{TR_{MRE}}\times \vec{SR_{MRE}}\\ ={\left[k\times t\times \vec{BR^{\prime }{}_{3}}-\vec{ND_{2}}\times t-\vec{OKE^{\prime }{}_{2}}\right]}^{\prime }+k\times \vec{BR_{MRE}}+k\times \vec{WR_{MRE}}\times \vec{LR_{MRE}}\\ +k\times \vec{TR_{MRE}}\times \left(\vec{TR_{MRE}}\times \vec{LR_{MRE}}\right)+2k\times \vec{TR_{MRE}}\times \vec{SR_{MRE}} \end{array}$$ (27)

From the above equation, it can be seen that the change approach and the intensity of change of representative manufacturing enterprises MRE has a significant positive effect on the change radical old and new dynamic energy conversion of other manufacturing enterprises in the industry.

Phase III manufacturing companies are

$$\vec{SR^{\prime }{}_{3}}=\frac{\vec{ND_{2}}\times t+\int_{t_{1}}^{t_{2}}\left(\vec{ND_{n}}+\vec{ND_{t}}+\vec{I_{l}}+\vec{I_{t}}+\vec{I_{n}}+\vec{I_{ok}}\right)}{e\times t}$$ (28)

$$\vec{BR^{\prime }{}_{3}}=\frac{\vec{ND_{2}}\times t+\vec{OKE^{\prime }{}_{2}}+\int_{t_{1}}^{t_{2}}\left(\vec{ND_{n}}+\vec{ND_{t}}+\vec{I_{l}}+\vec{I_{t}}+\vec{I_{n}}+\vec{I_{ok}}\right)}{t}$$ (29)

At this time, the value of $\vec{OKE^{\prime }{}_{2}}$ is negligible, therefore $\vec{SR^{\prime }{}_{3}}\approx \vec{BR^{\prime }{}_{3}}$, It can be seen that the third stage of strategic change and behavioral model change are of equal strength, and the two together maintain the new dynamic energy of green transformation of manufacturing enterprises to overcome the original old dynamic energy until the old dynamic energy is completely replaced, and then the process continues to cycle.

## 4. Analysis of calculation cases

### 4.1. Simulation of the old and new dynamics of manufacturing enterprises

Manufacturing company Z was selected for the example analysis with the following data: set; k = 498.9; K = 1003.49; phase period *T* ≈ 6; *θ*_2_ = 11°; Ω_2_ = 30°; *φ* = 25.628*rad*/*s*; *t* = 2; *δ*_4_ = 12°; *δ*_1_ = 23°; The second stage of MRE has : $\vec{SR_{MRE}}$ = 179.5035 $\vec{SR_{MRE}}=179.5035$; $\vec{BR_{MRE}}=166.432$.

As can be seen from Fig 3, manufacturing companies in the first stage, the incremental change approach is dominant, and with the deepening of the degree of incremental change, the old dynamic energy momentum increases, but with 180 as the turning point, after which the old dynamic energy momentum gradually becomes smaller with the further strengthening of incremental change and gradually loses its effect. As can be seen from Fig 4, the overall new momentum of manufacturing companies in the first stage does not change significantly with the increase in the overall level of the intensity of incremental change, and the overall level of new momentum does not increase significantly. But the intensity of incremental change has a relatively large increase in new momentum in this interval segment, followed by a sharp decrease in new momentum momentum decrease. The possible reason for this is that it shows that there is a more obvious conflict between old and new dynamic energy conversion in the process of progressive change in this stage of manufacturing enterprises, but the new dynamic energy momentum fails to overcome the old dynamic energy inertia, and this stage still has a positive effect on the transformation and upgrading of manufacturing enterprises through the improvement of the old dynamic energy.

**Fig 3:** The old dynamic energy change whit the progressive change of manufacturing enterprises in the first stage.

**Fig 4:** The new dynamic energy change whit the progressive change of manufacturing enterprises in the first stage.

As can be seen from Fig 5, in the second stage, there is a significant increase in the new momentum momentum of manufacturing firms, and both incremental and radical changes play different degrees of roles in this process, respectively. As can be seen from the above figure, until the intensity of change reaches 100, the growth of new momentum with radical change is faster than the growth of new momentum brought by incremental change, after which the market new momentum brought by incremental change After that, the growth rate of new dynamic energy from incremental change exceeds the increase of new dynamic energy from radical change. The possible reason is that manufacturing companies initially rely on radical innovation to attract market attention in order to gain a certain market share and market position, and open up niche markets outside the mainstream market through new, different and unique forms of products and services, after which the degree and intensity of product and service changes slow down again. As can be seen from Fig 6, the radical change in the process of increasing the new momentum of resources of manufacturing enterprises is more obvious than the role of gradual change.

**Fig 5:** The change trend of new dynamic energy of manufacturing enterprises in the second stage with different levels of change.

**Fig 6:** The change trend of new dynamic energy of manufacturing enterprises in the second stage with the degree of change.

As can be seen from Fig 7, in the third stage, new dynamic energy gradually replaces old dynamic energy, and progressive change and radical change work together, reflecting the "two-wheel drive" effect, and the new dynamic energy of manufacturing enterprises shows an obvious phenomenon of steady increase under the joint action of two types of change.

**Fig 7:** The change trend of new dynamic energy of manufacturing enterprises in the second stage with the change in different ways.

### 4.2. Analysis of the mechanism of overcoming the inertia of the old dynamic energy in the second phase of Z manufacturing enterprises

According to the study of inertia forces in theoretical mechanics, this paper further proposes that $\vec{I_{G}}$ represents the consistent inertia that manufacturing enterprise G needs to make in order to keep pace with the development of MRE’s old and new dynamic energy transition, by the incremental change inertia $\vec{I_{l}}$, radical change inertia $\vec{I_{t}}$ and conceptual change inertia $\vec{I_{n}}$, (let the effective resource set of manufacturing enterprise G be measured by 10,000 yuan), in order to get the incremental change inertia size $\vec{LI_{l}}$, radical change inertia size $\vec{LI_{t}}$, and conceptual change inertia size $\vec{LI_{n}}$, quantify how the change inertia overcomes the old dynamic inertia in the second stage of the old and new dynamic energy alternation process of manufacturing enterprises. According to the formula in Table 2, we can get

$$\vec{LI_{l}}=k\times \vec{LRB_{c}}=-k\times \left({\text{sin}}^{2}\;\theta_{2}-\text{cos}\;\Omega_{2}\right)=530.462$$ (30)

$$\vec{LI_{t}}=k\times \vec{LWR_{MRE}}\times \vec{LSR_{MRE}}=6780.71$$ (31)

$$\vec{LI_{n}}=k\times \vec{TR_{MRE}}\times \left(\vec{TR_{MRE}}\times \left(\vec{LSR_{MRE}}+\vec{LBR_{MRE}}\right)\right)=1249.644$$ (32)

$\vec{LI_{ok}}$ represents the size of the organizational inertia that needs to be changed when manufacturing company A is out of sync with the MRE technology development -—The size of the non-conforming inertia is the size of the old dynamic inertia. Based on the dynamic motion relationship, it is calculated that

$$\vec{LI_{ok}}=2k\times \vec{TR_{MRE}}\times \vec{LSR_{MRE}}=1178.072$$ (33)

According to the above calculation results, it can be seen that manufacturing enterprise Z in the second stage of the old and new dynamic energy conversion in order to overcome the old dynamic energy inertia that increased in the first stage of the initial change, the adoption of more radical changes and internal structural changes, this change affects the organization’s original interest structure and interest relations, the original manufacturing enterprise old dynamic energy can produce an effective blow.

## 5. Conclusions and recommendations

### 5.1. Research conclusion

(1) As a special manifestation of manufacturing transformation and upgrading, the green transformation of manufacturing industry, from the analysis of internal mechanism, has the alternation of old and new dynamic energy in its transformation process, and its old and new dynamic energy transformation has great consistency with the interaction between variables of energy transfer dynamic theory in physics. Based on the dynamic theory, with MRE as the center of mass, a representative enterprise G as the reference object of other enterprises within the manufacturing industry, and an enterprise in the industry as an arbitrary mass point of the mass point group, the motion of the mass point in an inertial system, a non-inertial system, is contrasted with the mechanism of the action of different degrees and aspects of change of the enterprise on the process of transformation of old and new dynamic energy. According to the second law of Newtonian mechanics and the momentum theorem, angular momentum theorem and dynamic energy theorem of the non-inertial system mass point group, the green transformation process is divided into three different stages: the first stage of the old dynamic energy dominates; the second stage of the old and new dynamic energy play a role together; the third stage of the new dynamic energy dominates.

(2) Comparing the old and new dynamic momentum change control relationship, it is found that the green transformation process of manufacturing enterprises involves a variety of variables, and the interaction relationship between variables in the green transformation process of manufacturing industry is simulated through the interaction relationship of forces in dynamic theory. The motion space constituted by the set of mass points and the space constituted by the group of manufacturing enterprises are compared in terms of the motion parameters of the center of mass, the parameter settings of the mass points, the inertia parameter settings of the change of mass points, the inertia parameter settings of the old dynamic energy of the mass points and the momentum parameter settings of the mass points, and the mechanical relations in theoretical mechanics reflect the change intensity, the momentum of the old dynamic energy, the strength and inertia of the new dynamic energy and the new dynamic energy in the process of the change of the old dynamic energy in the manufacturing industry. The interaction relationship between the old momentum, the new momentum and inertia in the process of old and new dynamic energy transition is reflected by the theoretical mechanics relationship, so as to construct a green transformation dynamic model of manufacturing industry.

(3) Manufacturing enterprises in the first stage of green transformation process did not implement obvious changes, the upgrading of manufacturing enterprises and the static system of theoretical mechanics corresponding to the stage of behavioral model change momentum change is greater than the strategic model change momentum change, in the first stage of manufacturing enterprises in favor of the old dynamic energy, the old dynamic energy through their own change optimization to strengthen its positive effect to adapt to the new requirements of upgrading changes in manufacturing enterprises. In the second stage, the stronger the strategic change ability of manufacturing enterprises, the greater the role of the new dynamic energy of production factors, and the change of representative enterprises in the industry plays an incentive and driving role for other manufacturing enterprises to implement changes, and the intensity of strategic change of manufacturing enterprises in this stage exceeds the intensity of behavioral change, and the frequency of strategic change of manufacturing enterprises is obviously higher than the frequency of behavioral change. In the third stage, the intensity of strategic change and the intensity of behavioral pattern change of manufacturing enterprises are equal, and the two together promote the conversion of old dynamic energy to new dynamic energy.

(4) By selecting Z manufacturing enterprises for simulation analysis, in the first stage, the incremental change approach is dominant, and the old dynamic energy momentum increases with the deepening of the change degree, and after increasing to 180, the old dynamic energy momentum shows a decreasing trend until it loses its effect. In this stage, the new dynamic energy did not change with the increase of incremental change intensity, and the overall trend was smooth, but when the change intensity reached, the new dynamic energy showed a substantial increase, and then dropped sharply. According to the analysis, the change was caused by the conflict between the old and new dynamic energy transformation. In the second stage, progressive change and radical change show different degrees of action, and the new momentum momentum of manufacturing enterprises increases significantly. Before the intensity of change reaches 100, the growth rate of new dynamic energy in the market of manufacturing enterprises with radical change is faster than that of progressive change, after which the growth rate of new dynamic energy in the market brought by progressive change exceeds that of radical change. In terms of the increase of new dynamic energy of manufacturing enterprises’ resources, the effect of radical change is more obvious than that of progressive change. In the third stage, the new dynamic energy gradually replaces the old dynamic energy, and the new dynamic energy of manufacturing enterprises shows a clear trend of steady increase due to the combined effect of progressive and radical changes.

(5) Through the analysis of the mechanism of overcoming the inertia of old dynamic energy in the second stage, it can be seen that in this stage, manufacturing enterprises are in a critical period of transformation and alternation of old and new dynamic energy, and the inertia of change promotes the replacement of old dynamic energy by new dynamic energy through overcoming the inertia of old dynamic energy, in which the inertia effect brought by conceptual change and radical change is more significant.

(6) Through the construction of manufacturing green transformation dynamic model, arithmetic simulation analysis, and old dynamic energy inertia overcoming mechanism analysis, as far as the overall change of manufacturing enterprises is concerned, strategic change and behavioral model change still play a key role in the process of green transformation of manufacturing enterprises.

(7) According to the model analysis, the green transformation of representative manufacturing enterprises in the industry plays a demonstration role in the transformation of other enterprises. Therefore, the government can support the green transformation of manufacturing enterprises by starting with representative manufacturing enterprises, actively encouraging them to take the lead in implementing changes and boldly promoting the transformation of old and new dynamics, so as to achieve the effect of other manufacturing enterprises in the industry following suit and catching up, forming a good learning-competition mechanism. The green transformation of manufacturing industry is essentially the rational allocation of production factors such as capital, labor and technology in the industry, and enterprises can take corresponding methods according to the stage they are in, for example, at the early stage of transformation, they can first carry out gradual change of the enterprise itself; in the middle stage of transformation focusing on the strategic change of the enterprise, they can first take radical change until the growth rate of new dynamic energy momentum of the enterprise slows down, and then take the gradual change method; in the late stage of transformation Strategic change and behavioral model change are carried out simultaneously.

### 5.2. Recommendations

When green transformation of manufacturing industry, not only external factors but also its own endogenous variables should be taken into consideration. The development dynamics of manufacturing industry within the industry is uneven and influenced by the development level and endogenous hindering factors, and most of the researches focus on the influence of exogenous environmental factors and ecological factors on the green transformation and upgrading of manufacturing industry, while ignoring the changes of the influence of endogenous variables on the green transformation, therefore, we should emphasize the absorption and summary of the research on the stages and evolution of the green transformation process of manufacturing industry, reasonably allocate the green transformation of manufacturing industry elements input, increase the financial investment in green transformation of manufacturing industry, improve the national support policy for green transformation of manufacturing industry, pay attention to and solve the influencing factors of high hindrance in green transformation of each manufacturing industry, the introduction of senior talents, the period of conversion and alternation of old and new dynamic energy, so as to achieve the purpose of accelerating the transformation of traditional manufacturing industry to green development.

(1) Cultivate the concept of green development and establish the awareness of low-carbon development. The strategic idea of sustainable development of green manufacturing transformation should be put in the primary position of manufacturing industry, accelerating the green transformation of manufacturing industry needs to form the manufacturing mode of saving resources and protecting environment, changing the traditional inefficient and low output inappropriate and environmental manufacturing production method, and actively creating the transformation system of resource-saving and environment-friendly green manufacturing industry with good efficiency. On the government side, actively implement the concept of green development, implement government subsidies and green reform preferential policies, build a platform to help enterprises gather capital, recruit talents and introduce technology, carry out cultural and creative activities, formulate green consumption policies, and use the Internet, media and social software to implant the concept of green consumption and low-carbon life into people’s hearts. In the manufacturing enterprises, the managers of manufacturing enterprises should strengthen their awareness of low-carbon development, formulate development strategies that take economic and environmental costs into account, and carry out targeted reforms in the process of transformation, taking into account market supply and demand and consumer preferences. In terms of commodity supply, while meeting consumer demand, enrich the green product categories, strictly control the quality of environmental products, reduce the price of green products, so that consumers prefer green and environmental goods.

(2) Establish a sound policy system for green transformation of manufacturing industry. In terms of policy formulation, the government should take into account regional differences, industry characteristics, the relationship between energy intensity and economic growth and other actual situations, and formulate targeted policy regulations, for example, adopting supervisory and control regulations for traditional high energy-consuming enterprises and regulatory and incentive mechanisms for innovative enterprises. In terms of policy implementation, through the development of implementation programs, setting established standards and evaluation programs, combined with government subsidized industrial policies, to stimulate the green transformation of manufacturing industries and remove barriers to policy implementation. In terms of policy supervision, green regulatory laws and regulations are formulated to clarify the subjects and scope of regulation. Develop energy consumption and pollution emission standards, improve public supervision and opinion feedback mechanisms, and form an open, fair, efficient and convenient regulatory system.

(3) Actively promote digital technology to empower the green transformation of manufacturing industry. From the viewpoint of its mechanism of action, digital empowerment mainly acts on the transformation of manufacturing enterprises through two aspects of scale effect and technology effect. The scale effect can be divided into its own scale effect and the scale effect of the region where the enterprise is located. In terms of its own scale effect, digital technology can improve the productivity of manufacturing enterprises by expanding the scale of production on the supply side and timely transmission of demand information, reducing energy use and investing more funds in green emission reduction, thus improving the level of pollution control of manufacturing enterprises. In terms of the scale effect of the region where the enterprises are located, digital technology can spatially cluster enterprises with strong ties or in close proximity to each other, accelerate information transfer and technology exchange among enterprises, thus promoting the external effects of knowledge and technology spillover from the clustered industries in the region, reducing enterprise input costs and improving enterprise productivity and energy utilization. In terms of technology effect, digital technology can improve energy utilization rate and advanced environmental protection equipment investment by enhancing manufacturing enterprises’ ability of technological progress and accelerating productive capital renewal of manufacturing enterprises, so as to realize green transformation of manufacturing enterprises.

(4) Establish a financial service guarantee system for the green transformation of manufacturing industry. The government takes the lead and financial institutions participate in actively developing green financial derivatives and innovating green financial products to reduce the risks borne by the green transformation of manufacturing industries due to low-carbon transformation. Create green financial institutions to provide preferential credit services for green transformation enterprises. At the same time, increase government policy support, lower loan interest rates and loan thresholds, provide transformation support funds for green transformation enterprises, build a green financial service trading platform, and reasonably deploy capital between manufacturing green transformation enterprises and all sectors of society.

(5) Strengthen the cooperation and exchange to promote the transformation and upgrading of manufacturing industry. There are differences in the level of green transformation of each manufacturing industry in the industry and the general environment in which it is located, so strengthen the exchange and cooperation of the manufacturing industry among the enterprises in the region, let some representatives of the green transformation of the enterprises in the industry play the role of leading the exchange, actively encourage and guide the exchange of the green transformation of the traditional manufacturing industry, boldly promote the transformation of the old and new dynamic energy in the green transformation of the manufacturing industry to achieve the transformation and upgrading of other manufacturing enterprises in the industry, and form a good The cooperation and exchange mechanism. In addition, strengthening the cooperation and exchange can not only promote the benign competition between the guiding manufacturing industries, but also help the development of green transformation of manufacturing industries between regions, so that the relevant industrial chain of green manufacturing industries can be better extended and the green transformation and upgrading of other manufacturing industries can be driven by the radiation effect of the leading manufacturing enterprises in the industry to achieve common development.

## 6. Limitations

This investigation has certain limitations. Although this paper researches the conversion of old and new dynamics in the green transformation process of manufacturing enterprises and analyzes the mechanism of the influence of endogenous dynamics in each stage of green transformation enterprises, however, it does not identify and distinguish the specific endogenous variable elements of enterprises and quantitatively analyze the mechanism of the influence of each element input, so it is still difficult for enterprises to identify the green transformation status and allocate resource elements in practice.

## 7. Future research

The further research direction in the future is to simulate the whole element structure of green transformation of manufacturing enterprises, combine qualitative and quantitative analysis of the influence mechanism between different green transformation element groups, provide quantitative identification tools for the state of green transformation of enterprises, provide specific strategy generation methods for green transformation, and provide guidance for the practice of green transformation of manufacturing enterprises.
